# Naloxone's Pentapeptide Binding Site on Filamin A Blocks Mu Opioid Receptor–Gs Coupling and CREB Activation of Acute Morphine

**DOI:** 10.1371/journal.pone.0004282

**Published:** 2009-01-27

**Authors:** Hoau-Yan Wang, Lindsay H. Burns

**Affiliations:** 1 Department of Physiology & Pharmacology, City University of New York Medical School, New York, New York, United States of America; 2 Pain Therapeutics, Inc., San Mateo, California, United States of America; University of Oldenburg, Germany

## Abstract

Chronic morphine causes the mu opioid receptor (MOR) to switch its coupling from Gi/o to Gs, resulting in excitatory signaling via both Gαs and its Gβγ dimer. Ultra-low-dose naloxone (NLX) prevents this switch and attenuates opioid tolerance and dependence. This protective effect is mediated via a high-affinity interaction of NLX to a pentapeptide region in c-terminal filamin A (FLNA), a scaffolding protein interacting with MOR. In organotypic striatal slice cultures, we now show that acute morphine induces a dose-dependent Go-to-Gs coupling switch at 5 and 15 min that resolves by 1 hr. The acute Gs coupling induced by 100 µM morphine was completely prevented by co-treatment with 100 pM NLX, (+)NLX, or naltrexone (NTX), or their pentapeptide binding site (FLNA_2561–2565_), which we show can act as a decoy for MOR or bind to FLNA itself. All of these co-treatments presumably prevent the MOR–FLNA interaction. Since ultra-low-dose NTX also attenuates the addictive properties of opioids, we assessed striatal cAMP production and CREB phosphorylation at S^133^. Correlating with the Gs coupling, acute morphine induced elevated cAMP levels and a several-fold increase in pS^133^CREB that were also completely blocked by NLX, NTX or the FLNA pentapeptide. We propose that acute, robust stimulation of MOR causes an interaction with FLNA that allows an initially transient MOR–Gs coupling, which recovers with receptor recycling but persists when MOR stimulation is repeated or prolonged. The complete prevention of this acute, morphine-induced MOR–Gs coupling by 100 pM NLX/NTX or 10 µM pentapeptide segment of FLNA further elucidates both MOR signaling and the mechanism of action of ultra-low-dose NLX or NTX in attenuating opioid tolerance, dependence and addictive potential.

## Introduction

Ultra-low-dose opioid antagonists have been shown to enhance opioid analgesia, minimize opioid tolerance and dependence [1], [2] and attenuate the addictive properties of opioids [3], [4]. Early electrophysiology data suggested that ultra-low-dose opioid antagonists block excitatory signaling of opioid receptors [1]. Chronic opioid-induced excitatory signaling is mediated by a switch in G protein coupling by MOR from Gi/o to Gs proteins [5], 6 and by stimulation of adenylyl cyclase II and IV by the Gβγ dimer [5], [7] originating from the MOR-associated Gs protein [8]. Ultra-low-dose NLX co-treatment suppresses opioid tolerance and dependence by preventing these MOR signaling alterations [5], and we recently identified the NLX binding site that mediates its protective effects as a pentapeptide segment in c-terminal FLNA [9].

A scaffolding protein best known for its actin-binding and cell motility function, FLNA also regulates cell signaling by interacting with a variety of receptors and signaling molecules [10], [11]. Onoprishvili et al. [12] first showed FLNA to interact with MOR and suggested a role in MOR downregulation and desensitization. Also implicating FLNA in desensitization, our recent organotypic striatal slice culture data showed that potentially disrupting the MOR–FLNA interaction via NLX's high-affinity binding to FLNA blocks the chronic morphine-induced G protein coupling switch by MOR [9]. Specifically, FLNA peptide fragments containing the NLX binding site blocked the protective effect of NLX on both the MOR–Gs coupling and downstream cAMP accumulation induced by chronic morphine (twice daily 1-hr exposures for 7 days), presumably by interfering with NLX's binding to FLNA in the tissues.

Again using organotypic striatal slice cultures, we show here that acute morphine causes a dose-dependent and transient MOR–Gs coupling that resolves by 1 hr. This is the first indication that MOR–Gs coupling occurs acutely and dynamically and is not only a consequence of chronic opioid treatment. To assess the involvement of FLNA in this acute opioid-induced Gs coupling, we co-treated slices with NLX, naltrexone (NTX), or FLNA_2561–2565_, their pentapeptide binding site, as a decoy for MOR. We also examined the effects of these treatments on cAMP production and downstream phosphorylation of the cAMP-response-element-binding protein (CREB) at S^133^ as a marker of addictive processes, since ultra-low-dose NTX attenuates the acute rewarding effects of opioids [3], [4]. CREB is activated by phosphorylation at S^133^ predominantly by protein kinase A (PKA) through binding of cAMP. Hence, increasing levels of cAMP from activation of adenylyl cyclase following MOR–Gs coupling could contribute to the acute rewarding or addictive properties of opiates. A partial mediation of the acute rewarding effects of opiates by Gs signaling could explain the apparent discrepancy that ultra-low-dose NLX or NTX can enhance opioid analgesia while also attenuating the addictive properties of opioids.

## Methods

### Animals

Male Sprague Dawley rats (200 to 250 g) purchased from Taconic (Germantown, NY) were housed two per cage and maintained on a regular 12-hr light/dark cycle in a climate-controlled room with food and water available *ad libitum.* For organotypic brain slice cultures, rats were sacrificed by rapid decapitation and striata were removed on ice and treated *in vitro* as described below. All procedures in this protocol are in compliance with the City College of New York IACUC on the use and care of animals.

### Organotypic striatal slice cultures

Rat brain slice organotypic culture methods were modified from those published previously [13], [14]. Striatal slices (200 µm thick) were prepared using a McIlwain tissue chopper (The Mickle Laboratory Engineering Co., Surrey, UK) at 4°C. Slices were immediately transferred to sterile, porous culture inserts (0.4 µm, Millicell-CM), using the rear end of a glass Pasteur pipette. Each culture insert unit contained 2 slices and was placed into one well of the 12-well culture tray. Each well contained 1.5 ml of culture medium composed of 50% MEM with Earl's salts, 2 mM L-glutamine, 25% Earl's balanced salt solution, 6.5 g/l D-glucose, 20% fetal bovine serum (FBS), 5% horse serum, 25 mM HEPES buffer and 50 mg/ml streptomycin and 50 mg/ml penicillin. The pH was adjusted to 7.2 with HEPES buffer. Cultures were first incubated for 2 days to minimize the impact of injury from slice preparation. Incubator settings were 36°C with 5% CO_2_.

### Determination of MOR–G protein coupling

To determine the dose-response of acute morphine on MOR–G protein coupling, slices were exposed to 0.1, 1, 10 or 100 µM morphine for 15 min. To assess the effect of ultra-low-dose NLX or NTX on the signaling switch induced by 100 µM morphine, some slices were exposed to 100 µM morphine plus 100 pM NLX or NTX. To determine whether NLX's effect may be mimicked by the site on FLNA that interacts with MOR, brain slices were incubated with morphine plus 10 µM VAKGL (FLNA_2561–2565_) or control pentapeptide, VAAGL. Peptides were purchased from Sigma-Genosys (The Woodlands, TX). A separate experiment was performed to assess the effect of 100 pM (+)NLX, the stereoisomer of NLX that is inactive at MOR. Slices were exposed to (+)NLX or (+)NLX plus 100 µM morphine for 15 and 60 min. Prior to treatments, culture medium was removed and the culture insert containing the slices was gently rinsed twice with warm (37°C) PBS (pH7.2) before incubation in 0.1% FBS-containing culture medium for 2 hr. Slices were transferred to fresh 0.1% FBS-containing culture medium with indicated agents. Tissues were harvested 5, 15 or 60 min after drug exposures by centrifugation. To determine of MOR–G protein coupling, slices were homogenated to generate synaptic membranes and cytosolic fractions. Synaptic membranes (400 µg) were solubilized with 0.5% digitonin/0.2% sodium cholate/0.5% NP-40 in 250 µl of immunoprecipitation buffer (25 mM HEPES, pH7.5; 200 mM NaCl, 1 mM EDTA, 50 µg/ml leupeptin, 10 µg/ml aprotinin, 2 µg/ml soybean trypsin inhibitor, 0.04 mM PMSF and a mixture of protein phosphatase inhibitors). Following centrifugation, striatal membrane lysates were immunoprecipitated with immobilized anti-Gαs/olf or -Gαo antibodies (Santa Cruz Biotechnology, Santa Cruz, CA) conjugated with immobilized protein A-agarose beads (Pierce-Endogen). The level of MOR in anti-Gαs/olf or -Gαo immunoprecipitates was determined by Western blotting using specific anti-MOR antibodies (Santa Cruz Biotechnology).

### Determination of cAMP accumulation

To measure the MOR-mediated increase in cAMP production, brain slices were incubated with Kreb's-Ringer (basal), 100 µM morphine and/or co-treatment with 100 pM NLX, NTX or 10 µM VAKGL (FLNA_2561–2565_ ) for 5, 15 and 60 min in the presence of 100 µM phosphodiesterase inhibitor, IBMX. For the 60-min timepoint, IBMX was added 15 min after morphine exposure. For the experiment that assesses cAMP production by Go-coupled MOR, slices were incubated with morphine, morphine plus 10 µM VAKGL, or 10 µM VAKGL for 5 or 60 min prior to incubation for 5 min with 10 µM forskolin. The reaction was terminated by placing slices in ice-cold Ca^2+^-free Kreb's-Ringer containing 0.1 mM EDTA and centrifugation. Tissues were homogenized by sonication and protein precipitated with 1M TCA and the supernatant obtained after centrifugation was neutralized using 500 mM Tris, pH9.0. The level of cAMP in brain lysates was measured by a cAMP assay kit (PerkinElmer Life Science, Boston) according to manufacturer's instructions.

### Determination of CREB activation

To assess whether acute high-dose morphine induces CREB activation and whether co-treatment with 100 pM NLX, NTX or the FLNA pentapeptide alter it, the level of protein kinase A-phosphorylated CREB, pS^133^-CREB, was assessed in cytosolic and nucleus fractions generated as described above from striatal slices. CREB in the solubilized cytosol and nucleus was immunoprecipitated with immobilized anti-CREB antibodies (Santa Cruz Biotechnology) and the level of pS^133^-CREB determined by Western blotting using a specific antibody directed against pS^133^-CREB (Santa Cruz Biotechnology).

Since CREB phosphorylation at the S^133^ can also be induced in response to elevated intracellular Ca^2+^, experiments were designed to assess the contribution of Ca^2+^ by including cell permeable intracellular Ca^2+^ chelator, BAPTA-AM. In this study, striatal slice cultures were treated with 100 µM BAPTA-AM for 30 min in serum-free medium prior to incubation with 100 µM morphine with or without 100 pM NLX, 100 pM NTX or 10 µM VAKGL pentapeptide. pS^133^-CREB levels in the solubilized cytosol and nucleus were measured as described above.

### Assessment of VAKGL peptide binding to MOR and FLNA proteins

To elucidate whether the pentapeptide FLNA fragment VAKGL functions as a MOR decoy by binding to MOR or interacts with full-length FLNA, we utilized a cell-free system. VAKGL biotinated at either n- or c-terminus (0.5 µg/well) was coated onto streptavidin-coated plates (Reacti-Bind^TM^ NeutrAvidin^TM^ High binding capacity coated 96-well plate, Pierce). Each condition had 12 replicates. After 3 washes with 200 µl PBS, immunoaffinity-purified FLNA (0.5 µg) from rat brain and A7 cells or MOR (0.1 µg) from rat brain or SK-N-MC cells were added into designated wells and incubation was carried out for 1 hr at 25°C with constant shaking. The plate was washed with PBS three times and the bound FLNA and MOR detected using anti-FLNA and -MOR antibodies followed by FITC-conjugated anti-mouse and -rabbit IgG, respectively. Following three washes with PBS, The FLNA and MOR signals were detected using a multi-mode plate reader (DTX-880, Beckman). The background FITC signal from matched wells, defined by the signal produced by unconjugated secondary antibodies at 100-fold higher dilution, was subtracted from the total signal. This background FITC signal was <15% of total signal in test wells.

### Data Analysis

All data are presented as mean±standard error of the mean. Treatment effects were evaluated by two-way ANOVA followed by Newman-Keuls test for multiple comparisons. Two-tailed Student's *t* test was used for *post hoc* pairwise comparisons. The threshold for significance was p<0.05.

## Results

### Acute morphine induces dose-dependent MOR–Gs coupling

After 15-min incubation with 0.1, 1, 10 or 100 µM morphine, some MOR–Gs coupling was noted in response to 0.1 µM morphine. With increasing dose, the Gs coupling progressively increased as the level of Go coupling decreased (Fig. 1). While a true comparison of the levels of Gs vs. Go coupling cannot be made since the antibodies detecting Gαs vs. Gαo may have different affinities, the progressive switch from Go to Gs coupling at 15 min of exposure to increasing doses of morphine is clearly visible. Additionally, although the anti-Gαs/olf antibody does not distinguish between these functionally similar Gs family members, the Gα protein detected here in striatum may be predominantly Golf[15].

**Figure 1:** Acute morphine causes a dose-dependent MOR – G protein coupling switch. Densitometric quantitation (*B*) of blots (*A*) shows that the level of MOR–Gs coupling after 15-min morphine exposure increases progressively as dose increases from 0.1 to 100 µM concentrations. In parallel, the level of MOR–Go coupling decreases with increasing morphine concentration. *n* = 4. *p<0.01 compared to respective Go or Gs/olf coupling of vehicle condition.

### Acute morphine-induced G protein coupling switch blocked by 100 pM NLX/NTX or 10 µM FLNA pentapeptide

An acute morphine-induced Go-to-Gs coupling switch in striatal slice cultures was blocked by co-exposure to 100 pM NLX or NTX or 10 µM concentration of their pentapeptide binding site on FLNA (Fig. 2). Morphine (100 µM) caused a complete Go-to-Gs coupling switch by MOR at 5 and 15 min of exposure. After 60 min of morphine exposure, the switch had resolved and no Gs coupling was detected. Co-treatment with 100 pM NLX or NTX prevented this acute G protein coupling switch by MOR (Fig. 2B). Similarly, pre-treatment with the pentapeptide binding site of NLX or NTX on FLNA (VAKGL; FLNA_2561–2565_) at 10 µM concentration also completely prevented this acute morphine-induced coupling switch by MOR (Fig. 2B). The control peptide, FLNA_2561–2565_ with one mid-point lysine-to-alanine substitution (VAAGL), did not prevent the MOR–Gs coupling, but mildly preserved Go coupling at 15 minutes. Exposure to NLX, NTX or either peptide alone without morphine had no effect on MOR coupling. In sum, the only significant differences compared to the vehicle condition for both Go and Gs coupling were the 5 and 15 minute timepoints for both morphine and morphine + the control peptide (VAAGL) (p<0.01 for each).

**Figure 2:** The Go-to-Gs coupling switch is transient and blocked by FLNA pentapeptide or 100 pM NLX/NTX. After 5, 15 or 60 min of drug treatment, striatal membranes were solubilized and immunoprecipitated with immobilized anti-Gα prior to detection with anti-MOR by Western blotting. Densitometric quantitation (*B*) of blots (*A*) shows the acute morphine-induced Go-to-Gs/olf coupling switch at 5 and 15 min timepoints that is prevented by co-treatment with 100 pM NLX or NTX or pre-treatment with the FLNA_2561–2565_ pentapeptide (VAKGL), but not the control pentapeptide (VAAGL). *n* = 4. *p<0.01 compared to respective Go or Gs/olf coupling of vehicle condition.

### (+)NLX also blocks acute morphine-induced MOR–Gs coupling

The naloxone isomer that is inactive as an opioid antagonist, (+)NLX, was used to confirm that the blockade of MOR–Gs coupling occurs by a mechanism other than antagonism of MOR. Similar to the blockade by a 100 pM concentration of the active isomer of NLX seen in Fig. 2, 100 pM (+)NLX blocked the Gs coupling induced by 15 min of 100 µM morphine (Fig. 3).

**Figure 3:** (+)NLX also blocked the transient Go-to-Gs coupling switch induced by acute high-dose morphine. After 15 or 60 min of drug treatment, striatal membranes were solubilized and immunoprecipitated with immobilized anti-Gα prior to detection with anti-MOR by Western blotting. Densitometric quantitation (*B*) of blots (*A*) shows that the inactive isomer of NLX, (+)NLX, blocks the acute morphine-induced Go-to-Gs coupling switch at 100 pM similar to NLX or NTX or pre-treatment with the VAKGL pentapeptide in fig. 2. *n* = 4. *p<0.01 compared to respective Go or Gs coupling of vehicle condition.

### NLX/NTX or the FLNA pentapeptide block acute morphine-induced cAMP production and CREB activation

Since 100 µM morphine induced a complete Go-to-Gs switch (Figs 1 and 2), we determined whether cAMP production is elevated in response. As expected, acute 100 µM morphine significantly increased cAMP levels at 5 and 15 min (Fig. 4A). This acute morphine effect was blocked by co-treatment with 100 pM NLX or NTX (Fig. 4A). Similarly, VAKGL but not the control peptide VAAGL at 10 µM concentration also completely prevented this acute morphine-induced cAMP elevation (Fig. 4A). Exposure to NLX, NTX or either peptide alone without morphine had no effect on cAMP levels. As with the morphine-induced Go-to-Gs switch, cAMP differed from vehicle control only for morphine and morphine+the control peptide (VAAGL) at the 5- and 15-min timepoints (p<0.01 for each). To demonstrate that MOR returns to Go coupling and inhibition of cAMP accumulation at 60 min, we performed a separate experiment using forskolin-stimulated cAMP production. With 10 µM forskolin added to each condition for 5 min, the inhibition of cAMP after 60 min of morphine exposure was visible (Fig. 4B), illustrating that the increased cAMP is not merely a result of desensitization of MOR with this high dose of morphine.

**Figure 4:** VAKGL or 100 pM NLX/NTX block an increased cAMP accumulation that parallels the coupling switch. *A*: Without stimulation by forskolin, the morphine-induced increase in cAMP accumulation was greatest in striatal slice cultures treated with morphine for 5 or 15 min but was still visible at 60 min. This increase was blocked by all co-treatments except the control peptide VAAGL. *B*: With forskolin stimulation, morphine increased cAMP accumulation at 15 min but decreased it at 60 min, indicating a reversion back to Go coupling. The VAKGL peptide again blocked the morphine-induced increase in cAMP accumulation. *n* = 4. **p<0.05; *p<0.01 compared to Kreb's-Ringer at the respective timepoint. #p<0.01 comparing VAKGL+morphine to morphine.

To further investigate this Gs-mediated activation of adenylyl cyclase by acute high-dose morphine (100 µM), we measured the potential downstream activation of CREB by its phosphorylation at serine-133. Morphine increased pS^133^CREB with a timecourse that paralleled that of the Gs coupling and cAMP accumulation (Fig. 5). A robust level of pS^133^CREB was detected in striatal tissue from slice cultures after 5 and 15 min of morphine exposure, while only a residual level was detected at 1 hr. Co-treatment with 100 pM NLX or NTX, or pre-treatment with 10 µM of the VAKGL pentapeptide, the binding site of NLX or NTX on FLNA (FLNA_2561–2565_), virtually abolished this signal. In contrast, pre-treatment with the control peptide VAAGL did not significantly diminish pS^133^CREB levels seen in the morphine only condition. Treatment alone with NLX, NTX or either peptide did not result in pS^133^CREB detection. Again, only morphine and morphine+the control peptide produced significant differences compared to the vehicle condition (p<0.01 for 5- and 15-min timepoints and p<0.05 for 60 min).

**Figure 5:** VAKGL or 100 pM NLX/NTX blocked the CREB activation induced by acute morphine. Densitometric quantitation (*B*) of Western blots (*A*) shows the activation of CREB, measured by pS^133^CREB detection, at 5 and 15 min of morphine exposure and its blockade by co-treatment with 100 pM NLX or NTX or pre-treatment with the VAKGL but not the VAAGL pentapeptide. *n* = 4. *p<0.01 and **p<0.05 compared to vehicle.

Because phosphorylation of CREB at S^133^ can also be achieved through elevation of Ca^2+^, we assessed the contribution of cAMP and Ca^2+^ to acute high-dose morphine-induced pS^133^CREB by inclusion of the cell permeable Ca^2+^ chelator, BAPTA-AM. Removal of Ca^2+^ did not affect the ability of morphine to increase pS^133^CREB or the blockade of this effect by NLX, NTX or VAKGL (Fig. 6). These data suggest that acute high-dose morphine increases pS^133^CREB mainly through the cAMP and protein kinase A pathway.

**Figure 6:** The calcium chelator BAPTA-AM did not notably diminish morphine-induced CREB activation or alter co-treatment effects. Densitometric quantitation (*B*) of Western blots (*A*) shows the activation of CREB, measured by pS^133^CREB detection, at 5 and 15 min of 100 µM morphine exposure and its blockade by co-treatment with 100 pM NLX or NTX or pre-treatment with the VAKGL but not the VAAGL pentapeptide. *n* = 4. *p<0.01 and **p<0.05 compared to vehicle.

### VAKGL binding to MOR or FLNA proteins

We last investigated whether the VAKGL pentapeptide is binding to MOR or full-length FLNA to prevent, in a manner similar to ultra-low-dose NLX, MOR's Gs coupling, the increased cAMP accumulation and the CREB activation following acute high-dose morphine. FLNA and MOR purified from two different sources each were tested for binding to VAKGL-coated plates and detected with anti-MOR or anti-FLNA antibodies followed by FITC-labelled secondary antibodies. Both MOR and FLNA bound VAKGL-coated plates (Fig. 7), suggesting that the VAKGL pentapeptide may disrupt the MOR–FLNA interaction by binding to MOR as a decoy for FLNA and/or by binding to FLNA itself.

**Figure 7:** The VAKGL pentapeptide binds both MOR and FLNA proteins. To assess the mechanism whereby FLNA_2561–2565_ pentapeptide (VAKGL) disrupts the MOR–Gs coupling, cAMP accumulation and CREB activation in a manner similar to 100 pM NLX or NTX, purified MOR and FLNA proteins were tested for binding to streptavidin-coated plates coated with biotinated VAKGL peptide. Both proteins, purified from two different sources, showed marked binding to the peptide, regardless of the peptide's orientation on the plate. The bound proteins were visualized with specific antibodies followed by FITC-conjugated secondary antibodies, and the background FITC signal from matched wells was subtracted from the total signal. *n* = 12.

## Discussion

Preferentially coupling to pertussis toxin-sensitive G proteins Gi and Go to inhibit the adenylyl cyclase/cAMP pathway (Laugwitz et al., 1993;Connor and Christie, 1999), MOR switches to Gs coupling after chronic opioid administration, resulting in excitatory signaling by both Gαs and Gβγ subunits [5], [6], [8]. Ultra-low-dose NLX co-treatment prevents this chronic opioid-induced G protein coupling switch and the instatement of Gβγ interacting with adenylyl cyclase, as well as the associated opioid tolerance and dependence [5]. Although the molecular pharmacology demonstrations of MOR–Gs coupling have used morphine, it is reasonable to assume that a variety of opioid agonists may similarly induce MOR–Gs coupling since ultra-low-dose NLX or NTX have been shown to enhance and prolong analgesia and prevent tolerance and dependence [1], [2], [16], [17], and attenuate addictive properties [3], [4] of oxycodone as well as morphine. While some level of Gs coupling has been previously detected in opioid-naïve or acute morphine exposed CHO cells [6], the present work in organotypic striatal slice cultures is the first to demonstrate that acute exposure to a high concentration of morphine causes predominant but transient MOR–Gs coupling similar to the persistent change following chronic morphine. This transient and dose-dependent G protein coupling switch of MORs, evident at 5 and 15 minutes of morphine exposure, is unlikely to represent an acute tolerance/dependence effect since MOR had completely reverted to its native Go coupling by 1 hour of morphine exposure. Instead we propose that with even this brief period of continued stimulation following high-dose morphine, MOR initially couples to Gs instead of Gi/o but is able to recover. With the repeated or prolonged MOR stimulation of chronic opiate exposure, however, this dynamic cycling from Gs back to Go evidently becomes impaired, leading to a persistent Gs coupling, behaviorally manifest as opioid analgesic tolerance and dependence.

Similar to ultra-low-dose NLX's suppression of the chronic morphine-induced coupling switch, the present data show that this acute morphine-induced coupling switch by MOR can be completely prevented by co-treatment with 100 pM NLX or NTX or 10 µM concentration of their pentapeptide binding site on FLNA. In addition, the equal efficacy in blocking this Gs coupling of 100 pM (+)NLX, the isomer that is inactive as an opioid antagonist, further confirms a mechanism of action other than antagonism of MOR. We previously discerned the precise binding site of NLX as FLNA_2561-2565_ using overlapping peptides and then blocked the protective effects of NLX on MOR–Gs coupling and cAMP accumulation in organotypic striatal slice cultures by co-incubation with decapeptides containing this binding site [9]. In this prior study, FLNA peptides presumably bound to NLX, blocking its prevention of the morphine-induced MOR–Gs coupling by preventing it from binding full-length FLNA in the tissues. These data led us to postulate that the interaction between MOR and FLNA, first demonstrated by Onoprishvili et al. (2003), was critical to the G protein coupling switch. We theorized that a particular FLNA–MOR interaction enables MOR to release from the signaling complex to couple to Gs upon subsequent receptor stimulation. In addition to FLNA, MOR has recently been shown to interact with another scaffolding protein, spinophilin (Charlton et al., 2008). While blocking the MOR–FLNA association, at least via ultra-low-dose NLX/NTX, diminishes tolerance, dependence and the rewarding effects of opiates, preserving or enhancing MOR's association with spinophilin appears to similarly modify these opioid effects.

In the present study, we showed the pentapeptide FLNA_2561–2565_ itself may act as a decoy for MOR to prevent the MOR–FLNA interaction and subsequent Gs coupling by MOR. This VAKGL pentapeptide was as effective as NLX or NTX as all three completely blocked the transient switch to Gs coupling by MOR during acute, high-dose morphine exposure. NLX and NTX presumably prevent the MOR–FLNA interaction by binding to their VAKGL binding site on FLNA, and this binding site on FLNA does appear be the approximate site on this protein that interacts with MOR. The demonstration that both purified MOR and FLNA proteins bind to VAKGL suggests that the VAKGL pentapeptide can similarly prevent the MOR–FLNA interaction but by binding to either protein. It is also possible that NLX and NTX block MOR–Gs coupling by changing the conformation of FLNA upon binding rather than by direct interference, and that by binding to “itself” in the full-length protein, VAKGL similarly prevents the changed FLNA conformation. Finally, since the VAKGL peptide can both prevent NLX's protective effects as in our prior study (Wang et al., 2008) as well as mimic NLX's protective effects when used alone in the current study, we theorize that this pentapeptide preferentially binds NLX but in its absence will interact with MOR or full-length FLNA. Further study is needed to elucidate the precise VAKGL interaction site on FLNA and MOR.

Our finding that all three co-treatments, NLX, NTX or the decoy pentapeptide also prevented morphine-induced CREB activation (as indicated by ser^133^ phosphorylation) in these striatal slice cultures may offer a mechanistic explanation for the attenuation of opioid reward and addictive processes by ultra-low-dose NTX. Found in all cells of the brain, CREB is a transcription factor implicated in addiction as well as learning and memory and several other experience-dependent, adaptive (or maladaptive) behaviors [18]. In general, CREB is inhibited by acute opioid treatment, an effect that is completely attenuated by chronic opioid treatment, and activated during opioid withdrawal [19]. However, a regional mapping study showed that opioid withdrawal activates CREB in locus coeruleus, nucleus accumbens and amygdala but inhibits CREB in lateral ventral tegemental area and dorsal raphe nucleus [20]. In the striatum, CREB activation has been viewed as a homeostatic adaptation, attenuating the acute rewarding effects of drugs [21], [22]. This view is supported by nucleus accumbens overexpression of CREB or a dominant-negative CREB mutant respectively reducing or increasing the rewarding effects of opioids in the conditioned place preference test [23]. In conflict, however, reducing nucleus accumbens CREB via antisense attenuated cocaine reinforcement as assessed in self-administration [24]. Clearly, CREB activation is implicated in addiction, but whether it directly contributes to the acute rewarding effects of drugs or initiates a homeostatic regulation thereof appears less clear.

Again, it is possible that the several-fold increase in pS^133^CREB observed here following acute, high-dose morphine might indicate acute dependence rather than acute rewarding effects; however, the transient nature of the MOR–Gs coupling and the return to inhibition of cAMP at 1 hr suggests otherwise. The correlation of pS^133^CREB with the MOR–Gs coupling and cAMP production following acute high-dose morphine exposure, as well as the similar treatment effects on all, suggest that this alternative signaling mode of MOR may contribute to the acute rewarding or addictive effects of opioids. This counterintuitive notion may explain the apparent paradox that ultra-low-dose NTX, while enhancing the analgesic effects of opioids, decreases the acute rewarding or addictive properties of morphine or oxycodone as measured in conditioned place preference or self-administration and reinstatement paradigms [3], [4]. If one considers analgesic tolerance, opioid dependence, and opioid addiction together as adaptive regulations to continued opioid exposure, a treatment that prevents MOR's signaling adaptation of switching its G protein partner may logically attenuate these seemingly divergent behavioral consequences of chronic opioid exposure. However, the acute rewarding effects of opioids are not completely blocked by ultra-low-dose opioid antagonists, suggesting that a MOR–Gs coupling may only partially contribute to the addictive or rewarding effects. Although ultra-low-dose NTX blocks the conditioned place preference to oxycodone or morphine [3], its co-self-administration only reduces the rewarding potency of these opioids but does not abolish self-administration outright [4]. Nevertheless, it is tempting to theorize that a direct stimulatory effect on VTA neurons, as opposed to the proposed disinhibition via inhibition of GABA interneurons [25], may play some role in opioid reward. Finally, a MOR–Gs coupling mediation of reward, increasing with increasing drug exposure, is in keeping with current theories that the escalation of drug use signifying drug dependence may not indicate a “tolerance” to rewarding effects but instead a sensitization to rewarding effects [26].

In summary, the present work has demonstrated that acute, high-dose morphine causes an immediate but transient switch in G protein coupling by MOR from Go to Gs similar to the persistent switch caused by chronic morphine. Ultra-low doses of NLX, NTX or even (+)NLX prevent this switch, just as ultra-low-dose NLX has previously been shown to attenuate the chronic morphine-induced coupling switch by MOR. The transient nature of this acute altered coupling suggests that in recycling, the receptor eventually recovers and couples to its native G protein. We hypothesize that with chronic opioid exposure, the receptor loses the ability to recover and continues to couple to Gs, activating the adenylyl cyclase/cAMP pathway, upregulating protein kinase A, and phosphorylating CREB as one downstream effector example. The persistently elevated phosphorylated CREB may then shape the expression of responsive genes including those closely related to drug addiction or withdrawal, such as brain-derived neurotrophic factor (BDNF)[27], and tolerance. Importantly, the equivalent blockade of Gs coupling and pS^133^CREB by the NLX and NTX pentapeptide binding site on FLNA further elucidates the mechanism of action of ultra-low-dose NLX and NTX in their varied effects. These data strengthen our hypothesis that a particular MOR–FLNA interaction allows MOR to couple to Gs and that disrupting this interaction, either by NLX/NTX binding to FLNA or via a FLNA peptide binding to MOR and/or FLNA, can prevent the altered coupling and attenuate tolerance, dependence and addictive properties associated with opioid drugs.
